The article "Multicentric paraspinal neuroglial heterotopia with Müllerian and renal agenesis: a variant of Mayer-Rokitansky-Küster-Hauser syndrome?" was published in 2013. Journal: Diagn Pathol.

# Multicentric paraspinal neuroglial heterotopia with Müllerian and renal agenesis: a variant of Mayer-Rokitansky-Küster-Hauser syndrome?

**DOI:** 10.1186/1746-1596-8-141

**Published:** 2013-08-22

**Authors:** Lu-Hau Deng, Chii-Hong Lee

**Affiliations:** 1 Department of Pathology, Taipei Medical University-Wan Fang Hospital, 111, Section 3, Hsing-Long Road, Taipei 11696, Taiwan; 2 Department of Pathology, Taipei Medical University-Shuang Ho Hospital, 291, Zhongzheng Road, Zhonghe District, New Taipei City 23561, Taiwan

**Keywords:** Neuroglial heterotopia, Müllerian agenesis, Renal agenesis, Mayer-Rokitansky-Küster-Hauser syndrome, Pathogenesis

## Abstract

**Abstract:**

Neuroglial heterotopia is a rare congenital anomaly that mostly involves the head and neck region. We report a female fetus with multicentric paraspinal neuroglial heterotopia in the retropharyngeal and retroperitoneal spaces, right renal agenesis, left renal hypoplasia, and Müllerian agenesis. Additional findings included bilateral preaxial polydactyly of the hands, megacystis, rectovesical fistula, and imperforate anus. The karyotype was 46, XX. This fetus had the features of Mayer-Rokitansky-Küster-Hauser (MRKH) syndrome with paraspinal neuroglial heterotopia. This is the first report of the co-occurrence of these two malformations which could share a common pathogenetic mechanism. We suggest this to be a variant MRKH syndrome.

**Virtual slides:**

The virtual slide(s) for this article can be found here: http://www.diagnosticpathology.diagnomx.eu/vs/3246922721015286.

## Introduction

Neuroglial heterotopia is a rare congenital anomaly that is probably related to neural tube defects [1-4]. It mostly affects the head and neck region, especially the nasal cavity. Only a few cases have been reported at other sites, such as the lungs [5] and retroperitoneum [2,6,7]. Multicentricity is exceptional [5], and concomitant congenital anomalies have not been reported in English literature. Here we present an unusual case of multicentric neuroglial heterotopia involving the retroperitoneal and retropharyngeal spaces accompanied by Müllerian agenesis, bilateral ovarian agenesis, right renal agenesis, left renal hypoplasia, rectovesical fistula, imperforate anus, and polydactyly.

## Case report

A 26-year-old female received regular prenatal care at our obstetric department during her second pregnancy. Oligohydramnios and fetal megacystis were detected by routine ultrasound at the 14th week of gestation. An amniocentesis test revealed a normal female 46, XX karyotype. The mother decided to terminate the pregnancy.

At autopsy, the female fetus weighed 85 g, and the crown-rump length was 12.2 cm. External examination revealed a typical phenotype of Potter sequence. Bilateral preaxial polydactyly of the hands was also noted. Internal examination revealed a disproportionately large urinary bladder, measuring 2.4 × 1.7 × 0.6 cm, accompanied by a rectovesical fistula and imperforate anus (Figure 1A). The left kidney was very small and weighed 0.02 g. The right kidney and bilateral ureters were not found. The bilateral ovaries and the müllerian structures, including the fallopian tubes, uterus, and vagina, were absent (Figure 1B). A white, soft and partially liquefied mass (2.8 × 2.2 cm) was found in the retroperitoneum (Figure 1A, 1B &1D). Another mass (1.5 × 1 cm) with a similar gross appearance was identified in the retropharyngeal space (Figure 1C &1D). The cranium and vertebral column were intact. No evidence of dorsal or ventral dysraphism or craniofacial defect was found. The leptomeninges were intact. The gross appearance of the brain and spinal cord was normal with autolysis.

The article "Multicentric paraspinal neuroglial heterotopia with Müllerian and renal agenesis: a variant of Mayer-Rokitansky-Küster-Hauser syndrome?" was published in 2013. Journal: Diagn Pathol.

**Figure 1:** **Internal examination in autopsy. (A &B)** Megacystis (asterisk), retroperitoneal neuroglial heterotopia (arrowhead), and uterine agenesis. **(C)** Retropharyngeal neuroglial heterotopia with autolysis (arrow). **(D)** Partially liquefied retroperitoneal and retropharyngeal neuroglial heterotopia after evisceration.

Histologically, both masses were composed of autolysed neuroglial tissue characterized by layers of cellular cortical plate and hypocellular white matter, resembling normal fetal cerebral tissue (Figure 2A &2B). Both the cortical plate and the white matter show positive immunoreactivity for CD56 and neuron-specific enolase (NSE) (Figure 2C). The glial tissue of the white matter was also positive for glial fibrillary acidic protein (GFAP) (Figure 2D). No other ectodermal, mesodermal or endodermal derivative was observed.

**Figure 2:** **Microscopic features of neuroglial heterotopia.** The retroperitoneal **(A)** and retropharyngeal **(B)** masses were composed of cellular cortical plate and hypocellular white matter. Both the cortical plate and the white matter were reactive for NSE **(C)** and the latter was also reactive for GFAP **(D)**.

## Discussion

Heterotopia, or choristoma, is applied to aggregates of normally formed tissues that are present in aberrant anatomical locations. Examples of heterotopias include a patch of gastric mucosa in the upper third of the esophagus, a rest of pancreatic tissue in the gastrointestinal wall, or a parathyroid gland within the thymus in the anterior mediastium. Heterotopia is usually an incidental finding, but it can be confused clinically with a neoplasm. In exceptional cases, true neoplasms may arise from heterotopic tissues [8,9].

The article "Multicentric paraspinal neuroglial heterotopia with Müllerian and renal agenesis: a variant of Mayer-Rokitansky-Küster-Hauser syndrome?" was published in 2013. Journal: Diagn Pathol.

Neuroglial heterotopia is a rare developmental anomaly with a rich variety of clinical features, pathological findings, and pathogenetic mechanisms. Based on anatomical location and pathological differentiation, Hori et al. proposed a classification of neuroglial heterotopia into extraneuraxial and paraneuraxial groups [2]. Extraneuraxial neuroglial heterotopia is much more common and usually involves the nasal cavity or the superficial soft tissue of the head and neck. Pathologically, it is characterized by a disorganized mixture of neuroglial and mesenchymal tissues or a lump of organized neural tissue similar to normal brain histology. It is often obvious at birth but may remain asymptomatic until late childhood or even adulthood. Complete surgical excision is curative in most cases [1,3,10,11]. On the other hand, paraneuraxial neuroglial heterotopia is rare and may involve the paracranial or paraspinal spaces, such as the occipital bone, retroperitoneum, and deep neck. It is composed of organized brain tissue and is usually diagnosed shortly after delivery or in early childhood. Disease-related complications are common [2,6,7,12,13].

The pathogenesis of neuroglial heterotopia is uncertain. Several pathogenetic hypotheses of extraneuraxial neuroglial heterotopia have been proposed, including (1) herniation of neuroectodermal tissue through a primary bony defect that is followed by a partial or complete secondary closure resulting in sequestration of the herniated tissue [1,3]; (2) separation and detachment of cerebral precursors (which later mature ectopically) from the brain primordium in early embryogenesis [1,12]; (3) aberrant migration of pluripotential embryonic tissue with subsequent neuroglial differentiation [1]; (4) retention of neuroectodermal remnants [14]; and (5) teratoma formation with a predominant or exclusive neuroglial component [1]. However, no single hypothesis can completely explain all the varieties of extraneuraxial neuroglial heterotopia. In contrast, paraneuraxial neuroglial heterotopia is closely related to neural tube defects, such as encephalocele and myelomeningocele. For instance, paraneuraxial neuroglial heterotopia shares a similar anatomical distribution and histological features with encephalocele and myelomeningocele [2,5-7,12,13]. A connection between the heterotopic neuroglial tissue and the intervertebral region via a string of connective tissue is found in some cases, and this gross picture is not much different from that of a myelomeningocele with an obliterated connection to the spinal cord [2,6]. Accordingly, the “herniation and sequestration” hypothesis seems tenable to explain the pathogenesis of paraneuraxial neuroglial heterotopia. The process of “herniation and sequestration” acts like a mild or “partially corrected” version of neural tube defects. This is probably why concomitant congenital anomaly is far less frequent in paraneuraxial neuroglial heterotopia than in encephalocele and myelomeningocele.

The article "Multicentric paraspinal neuroglial heterotopia with Müllerian and renal agenesis: a variant of Mayer-Rokitansky-Küster-Hauser syndrome?" was published in 2013. Journal: Diagn Pathol.

In this report, we present a case of multifocal paraneuraxial, paraspinal neuroglial heterotopia concomitant with congenital anomalies associated with Mayer-Rokitansky-Küster-Hauser (MRKH) syndrome. MRKH syndrome is regarded as an inhibitory malformation of the Müllerian ducts. It is characterized by agenesis of the uterus and the upper two-thirds of the vagina in individuals with a normal female karyotype [15,16]. Associated anomalies of the renal, skeletal and cardiovascular systems are present in about half of cases, and this severe form of the disease is categorized as atypical MRKH or MURCS association [15,16]. Ovarian agenesis, imperforated anus, polydactyly, and encephalocele have also been reported [15-18]. Although the pathogenesis of MRKH syndrome remains unclear, it is suggested that the spectrum of anomalies are attributed to the extent of developmental field defects that primarily affect the fetal mesoderm or its progenitor tissue in early embryogenesis [16]. When such mesodermal defects involve the paraaxial mesoderm, encephalocele, myelomeningocele and paraneuraxial neuroglial heterotopia may develop [1,3,19]. Given the similarity of the pathogenetic hypotheses for paraspinal neuroglial heterotopia and Müllerian agenesis, we suggest that the present case constitutes an unusual variant of MRKH syndrome.

## Consent

Written informed consent was obtained from the parent of the fetus for the use of the images and case presentation for educational and scientific purposes provided the unique personal identification is not revealed.

## Competing interests

Both authors declare that they have no competing interests.

## Authors’ contributions

LHD prepared this case report and literature review. CHL is the attending pathologist who performed the autopsy, made the diagnosis and finalized the manuscript. Both authors read and approved the final manuscript.
